# Influence Factors and Predictive Models for the Outcome of Patients with Ischemic Stroke after Intravenous Thrombolysis: A Multicenter Retrospective Cohort Study

This article has been retracted.

**DOI:** 10.1155/2022/3363735

**Published:** 2022-08-17

**Authors:** Jin Hu, Zhixian Fang, Xia Lu, Fei Wang, Ningyuan Zhang, Wenliang Pan, Xinzheng Fu, Gongchun Huang, Xiaoli Tan, Wenyu Chen

**Affiliations:** ^1^Department of Neurology, The Affiliated Hospital of Jiaxing University, Jiaxing, China; ^2^Department of Respiration, The Affiliated Hospital of Jiaxing University, Jiaxing, China; ^3^Department of Neurology, The First People's Hospital of Jiashan County, Jiaxing, China; ^4^Department of Neurology, The First People's Hospital of Tongxiang, Jiaxing, China; ^5^Department of Neurology, The People's Hospital of Haiyan, Jiaxing, China; ^6^Department of Neurology, The People's Hospital of Haining, Jiaxing, China; ^7^Department of Neurology, The First People's Hospital of Pinghu, Jiaxing, China

## Abstract

**Objective:**

Intravenous thrombolysis (IVT) is currently the main effective treatment for patients with ischemic stroke. This study aimed to analyze the factors affecting the early neurological recovery and prognosis of thrombolytic therapy after surgery and to construct predictive models.

**Materials and Methods:**

A total of 849 patients with ischemic stroke who received IVT treatment at six centers from June 2017 to March 2021 were included. Patients were divided into the training cohort and the validation cohort. Based on the independent factors that influence the early recovery of neurological function and the prognosis, the respective predictive nomograms were established. The predictive accuracy and discrimination ability of the nomograms were evaluated by ROC and calibration curve, while the decision curve and clinical impact curve were adopted to evaluate the clinical applicability of the nomograms.

**Results:**

The nomogram constructed based on the factors affecting the prognosis in 3 months had ideal accuracy as the AUC (95% CI) was 0.901 (0.874~0.927) in the training cohort and 0.877 (0.826~0.929) in the validation cohort. The accuracy of the nomogram is required to be improved, since the AUC (95% CI) of the training cohort and the validation cohort was 0.641 (0.597~0.685) and 0.627 (0.559~0.696), respectively.

**Conclusions:**

Based on this ideal and practical prediction model, we can early identify and actively intervene in patients with ischemic stroke after IVT to improve their prognosis. Nevertheless, the accuracy of predicting nomograms for the recovery of early neurological function after IVT still needs improvement.

## 1. Introduction

The Global Burden of Diseases, Injuries, and Risk Factors (GBD) study estimates rank stroke as the second most common cause of death in the world [1, 2] and the third most common cause of disability-adjusted life years (DALYs) [3], with 75% of stroke deaths and 81% of disability-adjusted life years occur in low- and middle-income countries [4]. Stroke can be divided into ischemic stroke and hemorrhagic stroke. Ischemic stroke is caused by the sudden loss of function led by the interruption of blood supply to part of the brain, and hemorrhagic stroke is caused by angiorrhexis or abnormal blood vessel structure [5]. In general, ischemic stroke accounts for about 80% of stroke cases, and hemorrhagic stroke accounts for about 20%, but the actual proportion of stroke types depends on different patients [6]. According to data from the Chinese Hospital Quality Monitoring System, in 2018, China's 1853 tertiary A hospitals admitted a total of 3,010,204 stroke inpatients, of which 2,466,785 were ischemic stroke patients, accounting for 81.9% [7]. On a global scale, the burden of stroke has increased significantly in the past few decades due to the increase in population size and aging population and the prevalence of changeable risk factors for stroke [8, 9]. Studies have shown that at the beginning of the twenty-first century, about 1.1 million Europeans suffer from stroke each year, and it is predicted that by 2025, 1.5 million Europeans will suffer from stroke each year, and the incidence of young people will gradually increase [10].

Acute reperfusion therapy is by far the most effective method for the treatment of patients with acute ischemic stroke [11]. However, after thrombolytic therapy, the early neurological function of a large number of patients has not been effectively improved. Some patients have poor prognosis after 90 days of treatment. The situation is not optimistic. This part of patients tends to bring an increasingly huge burden to the family and society [12]. This study aims to analyze the factors affecting the early neurological function of patients with acute ischemic stroke (intravenous thrombolysis, IVT) and the prognosis at 3 months after surgery and to establish a predictive model to improve the safety and effectiveness of thrombolytic therapy.

## 2. Materials and Methods

We included ischemic stroke patients undergoing IVT treatment from six centers (the First People's Hospital of Pinghu, the First Hospital of Jiaxing, the First People's Hospital of Jiashan, the First People's Hospital of Tongxiang, the People's Hospital of Haiyan, and the People's Hospital of Haining from June 2017 to March 2021). According to the inclusion and exclusion criteria, the cases that fit this study were selected.

The inclusion criteria are as follows: (1) 18 years old or older; (2) patients treated with alteplase thrombolysis and whose symptom onset time (referring to the time from symptom onset to thrombolytic treatment) ≤ 4.5 hours, while patients treated with urokinase and whose symptom onset time ≤ 6 hours; (3) cerebral infarction is diagnosed, and there is a certain neurological deficit; and (4) the patient or his family members agree to sign an informed consent.

The exclusion criteria are as follows: (1) patients with hemorrhagic cerebral infarction; (2) patients with transient ischemic attack; (3) patients with cerebral venous sinus thrombosis; (4) patients with brain tumors; (5) patients whose main observation indicators are incomplete due to various reasons; and (6) patients with contraindications to IVT (such as intracranial hemorrhage, history of intracranial hemorrhage, intracranial tumor, giant intracranial aneurysm, active visceral hemorrhage, platelets less than 100◊109/L, oral anticoagulant and INR> 1.7 or PT> 15 seconds, and intracranial or intraspinal surgery within 3 months before IVT).

### 2.1. Patient and Public Involvement

No patient was involved

### 2.2. Data Collection and Prognosis Classification

The data collected in this study were mainly patient baseline data and outcome indicators, including general information (gender, age, BMI, NIHSS score at admission, and smoking), some past medical history (secondary thrombolysis, hypertension, previous atrial fibrillation and previous ischemic heart disease, etc.), previous medication history (aspirin, clopidogrel, warfarin, atorvastatin, and rosuvastatin), laboratory test results (systolic pressure before thrombolysis, diastolic pressure before thrombolysis, hemoglobin, red blood cell count, etc.), treatment information (thrombolysis time and thrombolytic medication), and outcome indicators (24-hour NIHSS score and mRS score at 3 months after surgery). This study discussed the early neurological function recovery after thrombolytic therapy and the prognosis at 3 months. Among them, the early recovery of neurological function was assessed by the National Institutes of Health Stroke Scale (NIHSS) [13], and the prognosis at 3 months after the operation was assessed by the modified Rankin scale. The specific groups are as follows:

1. Early neurological function recovery [14]. *δ* ≥ 4 or 24-hour NIHSS≤1 was defined as the good early neurological function recovery group (group 0), and *δ* < 4 and 24-hour NIHSS>1 was the poor early neurological function recovery group (group 1). Besides, *δ* = NIHSS at admission 24-hour NIHSS
2. Prognosis at 3 months after surgery [15]. The prognosis at 3 months after surgery was measured by mRS score at 3 months after surgery, and the specific definition is as follows: mRS score at 3 months after surgery ≤2 was defined as the good prognosis group (group 0), and mRS score> 2 at 3 months after surgery was considered as the short-term poor prognosis group (group 1).

### 2.3. Model Construction and Verification

The samples included in this study were divided into training cohorts and verification cohorts at a ratio of 7 : 3 by nonrepeated random sampling. Variables with *P* < 0.1 based on the univariate analysis in the training cohort were used as predictors [16] and included them in the multivariate binary logistic regression. The entry method was Forward: LR. Then we analyzed the independent influencing factors that affected the early recovery of neurological function and the prognosis at 3 months after the surgery and established the predictive nomograms, respectively. In the training cohort and verification cohort, ROC curve and calibration curve were used to evaluate the predictive accuracy and discrimination ability of the nomogram, and the decision curve analysis (DCA) and clinical impact curve analysis (CICA) were used to evaluate the nomogram and the clinical applicability of [17, 18].

### 2.4. Statistical Analysis

SPSS 23 statistical software (IBM, Armonk, NY) was used to support univariate analysis and multivariate binary logistic. Continuous data is demonstrated as mean ± standard deviation or median (lower quartile and upper quartile), and *t*-test or Mann–Whitney *U* test was used for the comparison between the two groups; categorical data was demonstrated as *n* (%), and the chi-square test was used for comparison between groups. The construction of the nomogram and the drawing of ROC, decision curve, and clinical impact curve were completed in R4.0.4. Bilateral *P* < 0.05 was considered statistically significant.

## 3. Results

### 3.1. Patient Information

We enrolled 1,318 stroke patients who received IVT treatment from six hospital centers from June 2017 to March 2021 and excluded patients with hemorrhagic stroke, transient cerebral ischemia, complemented main indicators, and contraindications to IVT, and finally 849 patients were included in this study. Among the samples, 452 patients had poor recovery of neurological function in the early stage, and 294 patients had a poor prognosis at 3 months postoperatively. We use nonrepetitive random sampling at a ratio of 7 : 3, and draw the training cohort (594 cases) and the verification cohort (255 cases). In the training cohort, 320 patients had poor recovery of early neurological function, and 209 patients had a poor prognosis at 3 months postoperatively. In the verification cohort, 132 patients had poor recovery of neurological function early, and 85 patients had poor prognosis at 3 months after surgery (Table 1 and Figure 1).

### 3.2. Prognosis Prediction Model at 3 Months after Surgery

#### 3.2.1. Univariate Analysis

The univariate analysis of the prognosis of patients with ischemic stroke at 3 months after IVT showed that gender, age, BMI, NIHSS score at admission (BNIHSS), smoking, hypertension, previous atrial fibrillation (preAF), new-onset atrial fibrillation (NewAF), congestive heart failure (CHF), previous stroke history (PreStrokeHistory), clopidogrel history (Clopidogrel), rosuvastatin history (Rosuvastatin), pre-thrombolysis systolic blood pressure (PreSBP), hemoglobin (Hb), red blood cell count (RBC), neutrophils (N), APTT, INR, fibrinogen (Fg), medication time (Time), thrombolytic medication (Drug), and 24-hour NIHSS score (24hNHISS) were significantly different between the two groups (*P* < 0.05). Although diabetes (DM) and PT were not significantly different between the two groups (*P* > 0.05), they were close to 0.05. The above factors may affect the prognosis of patients with ischemic stroke at 3 months after IVT (Table 2).

### 3.3. Model Construction

The above-mentioned possible influencing factors were used as independent variables, and the prognosis at 3 months after IVT was used as the dependent variable. Multivariate binary logistic regression analysis was used, and the Forward: LR was used as the independent variable entry method. We analyzed the independent influencing factors that affect the prognosis of patients with ischemic stroke at 3 months after IVT. The analysis results show that age, diabetes DM, APTT, thrombolytic medication (Drug), and 24-hour NIHSS score (24hNIHSS) were independent factors influencing the prognosis of patients with ischemic stroke at 3 months after IVT, and a nomogram of the prognosis was constructed (Table 3).

#### 3.3.1. Model Verification

The accuracy of the nomogram predicting the prognosis at 3 months after IVT was analyzed by the ROC curve, and the AUC (95% CI) in the training cohort was 0.901 (0.874~0.927), the AUC in the verification cohort (95% CI) is 0.877 (0.826~0.929), which shows that the prognosis at 3 months after surgery can be well predicted. The calibration curve based on the training and verification cohort shows that the predicted value of the nomogram for the poor prognosis is in good accordance with the actual value (Figure 2).

Decision curve analysis (DCA) and clinical impact curve analysis (CICA) were used to evaluate the clinical applicability of nomogram predicting the prognosis of patients with ischemic stroke at 3 months after IVT. Both showed that the model had a large practical threshold probability range Pt> 0.3, and the benefit was higher. The figure showed that when the threshold probability Pt = 0.4, the cost/benefit = 2 : 3. CICA hypothesized that if the prognosis of 1000 people was evaluated, and we compared the model evaluation results with the actual results, when Pt = 0.4, the two curves came to be very close (that is, the number of high-risk patients predicted by the model was very close to the actual number of high-risk patients). In summary, this model had a very ideal effect on the prognosis of 3 months after IVT (Figure 3).

### 3.4. Predictive Model of Early Neurological Function Recovery

#### 3.4.1. Univariate Analysis

The results of univariate analysis of the early recovery of neurological function of patients with ischemic stroke after IVT showed that age, BMI, NIHSS score at admission (BNIHSS), hypertension, previous atrial fibrillation (preAF), diabetes (DM), systolic blood pressure before thrombolysis (PreSBP), red blood cell count (RBC), neutrophils (N%), APTT, treatment time ONT (Time), and thrombolytic medication (Drug) were significantly different between the two groups (*P* < 0.05), although gender, second thrombolysis (SecondThrombolysis), and fibrinogen (FG) are not significantly different (*P* > 0.05) but less than 0.1. The above factors may be the influencing factors of early neurological function after IVT in patients with ischemic stroke (Table 4).

#### 3.4.2. Model Construction

The above-mentioned possible influencing factors were used as independent variables, and the early neurological function recovery after IVT was used as the dependent variable. Multivariate binary logistic regression analysis was used, and the Forward: LR was used as the independent variable entry method. We analyzed the independent factors affecting the early recovery of neurological function in patients with ischemic stroke after IVT. The analysis results showed that age, NIHSS score at admission (BNIHSS), diabetes (DM), neutrophils (N), and medication (Drugs) were independent factors affecting the prognosis of IVT patients with ischemic stroke, and a nomogram of the prognosis was constructed (Table 5).

#### 3.4.3. Model Verification

The accuracy of the nomogram for early neurological function prediction was analyzed by ROC curve. The AUC (95% CI) in the training cohort was 0.641 (0.597~0.685), and the AUC (95% CI) in the verification cohort was 0.627 (0.559~0.696), which showed that the effect of distinguishing early neurological function was not ideal. The calibration curve based on the training cohort and the validation cohort showed that the predicted value of the nomogram for poor prognosis was in good accordance with the actual value (Figure 4).

Decision curve analysis (DCA) and clinical impact curve analysis (CICA) were used to evaluate the clinical applicability of the nomogram predicting early neurological recovery. Both showed that the model had a relatively narrow range of practical thresholds. CICA hypothesized that if the prognosis of 1000 people was evaluated, and we compared the model evaluation results with the actual results, when Pt> 0.6, the two curves came to be very close (that is, the number of high-risk patients predicted by the model was very close to the actual number of high-risk patients). At this time the cost/benefit = 3 : 2 (Figure 5).

## 4. Discussions

At present, there are a variety of effective treatment for patients with acute ischemic stroke, such as IVT and intravascular interventional therapy, which can improve the neurological outcome of patients, and the two can be combined for appropriate patients [19, 20]. But still, IVT is still the first choice for a large number of patients. The China Stroke Prevention and Treatment Report 2019 shows that the number of people receiving IVT treatment in 298 advanced stroke centers in China in 2018 was 43,486 [21, 22]. Not all patients can benefit from thrombolysis. A study by Emberson et al. showed that 69% of patients still had a poor prognosis (mRS ≥ 3 points) at 3 months after thrombolysis [23]. Poor prognosis not only reduces the direct benefits of IVT, but also reduces the quality of life of patients and increases the medical burden on the family and society [24]. The results of the ECASS III test shows that IVT at 3.0-4.5 h still has effect [25], and the IST-3 test shows that IVT on the onset of disease within 6 hours have effect [26]. The subjects of this study were enrolled from six centers who received IVT treatment within 6 hours of acute ischemic stroke since the onset of the disease. This study discusses and analyzes the factors affecting the early neurological function recovery after IVT and the prognosis at 3 months after the surgery and establishes corresponding prediction model to form an early identification and active intervention of patients who may have a poor prognosis and improve their prognosis.

This study shows that old age, diabetes, and urokinase thrombolysis are risk factors for poor early recovery of neurological function and poor prognosis at 3 months after IVT in patients with ischemic stroke. Guidelines for the primary prevention of stroke point out that [27] old age and diabetes are not only independent risk factors for the occurrence of acute ischemic stroke, but are also considered to be important risk factors affecting the prognosis of IVT. Older age is one of the most important and independent predictors of stroke death and adverse outcomes [28, 29]. A study by Ulrich et al. [30] showed that diabetes more than doubled the risk of stroke. About 20% of diabetic patients die of stroke. The course of diabetes also increases the risk of nonhemorrhagic stroke. Morgenstern et al. [31] verified that age-specific incidence and rate showed that diabetes would increase the incidence of ischemic stroke in all age groups. The thrombolytic stroke prediction model incorporates age and diabetes history into the predictive variables. The model has an ideal effect in predicting the prognosis of thrombolytic therapy for good and severe prognosis (*C* values are 0.79 and 0.78, respectively) [32]. In recent years, recombinant tissue-type plasminogen activator (rt-PA) has been approved by the US Food and Drug Administration (FDA) and European Medicines Agency (EMEA) as the only thrombolytic drug that can be used for ischemic stroke. However, due to the high cost, extremely short treatment window, and increased risk of bleeding if out of the treatment window, a large number of ischemic stroke patients worldwide have not benefited from the drug. Urokinase plasminogen activator (u-PA) is usually used as an alternative [33]. As mentioned above, among the 43,486 patients in China in 2018, 7282 patients were treated with urokinase thrombolysis, accounting for 16.7%, and the rest were treated with rt-PA. A nationwide prospective Chinese registry study with a sample size of 3810 [34] compared the efficacy of rt-PA and u-PA in ischemic stroke. The results showed that the two treatments have an excellent outcome (90-day mRS; there was no significant difference between score< 2) and symptomatic bleeding (*P* > 0.05). This study showed that compared with rt-PA, u-PA can significantly increase the risk of poor early neurological function recovery and poor prognosis at 3 months after surgery.

In addition, this study shows that the NIHSS score at admission and the proportion of centrifugal cells before thrombolysis are also independent factors influencing the poor early of neurological function recovery after IVT. Perez-de-Puig et al. [35] showed through animal experiments that the accumulation of neutrophils can cause the destruction of the blood-brain barrier, thereby increasing the risk of hemorrhagic transformation and the incidence of poor prognosis after IVT. The clinical study of Liu et al. [36] showed that the increase in neutrophil count and neutrophil percentage before thrombolysis is associated with an increased risk of poor prognosis in patients with ischemic stroke after IVT. The NIHSS score at admission is used as a scale for the severity of stroke, and the severity of the disease is positively correlated with its score. Therefore, a large number of predictive models for the prognosis of thrombolysis included NIHSS score at admission as a variable [37].

At the same time, the NIHSS score 24 hours after thrombolysis and APTT before thrombolysis are also independent factors influencing the prognosis at 3 months after IVT. This study showed that the NIHSS score 24 hours after IVT is an independent influencing factor of the prognosis at 3 months after surgery rather than the NIHSS score at admission. This shows that the severity of the disease after IVT can better predict the prognosis at 3 months postoperatively than the severity before treatment. Rangaraju et al. [38] verified that the NIHSS score at 24 hours in the postmortem analysis of 2 randomized controlled stroke trials can better predict the long-term outcome of ischemic stroke. Yongtao et al. [39] showed that APTT level before thrombolysis is an independent risk factor that influences the early neurological improvement of acute ischemic stroke after intravenous IVT. APTT prediction of the best segmentation point of early neurological function improvement before thrombolysis is at 27.15(s). When the APTT level is <27.15(s), the early neurological function improvement is significantly better than APTT>27.15(s). However, the relationship with the prognosis at 3 months after IVT has not been verified.

In recent years, the relationship between smoking and adverse outcomes after IVT for ischemic stroke has not yet been confirmed. The study of Moulin et al. [40] showed that smoking does not independently affect the prognosis of patients with cerebral ischemia treated with rt-PA. The better outcome of smokers is the result of different case combinations. This is also verified by the study of Kurmann et al. [41]. In the study of Sun et al. [42], smoking increases the risk of hemorrhagic transformation (HT) after IVT. This study shows that smoking is not an independent factor influencing the prognosis of IVT in patients with ischemic stroke. And among smoking patients, the propensity scoring method was used to match patients with high smoking age (>30 years) and patients with low smoking age (≤30 years), and it is found that the poor prognosis of the two was also very similar (see Table S1 and Table S2).

### 4.1. Limitations

This study has certain limitations. Although the factors that affect the early recovery of neurological function after IVT have been analyzed, the accuracy of the prediction nomogram for the recovery of early neurological function established based on this needs to be improved.

## 5. Conclusions

This study uses only a small number of indicators to establish a predictive model for the early neurological recovery of patients with ischemic after IVT and the prognosis at 3 months after surgery. These predictive factors are easy to obtain in clinical practice. There is a large difference in the prediction accuracy of the two models (Delong's test *P* < 0.05). The accuracy of the prediction nomogram based on the recovery of early neurological function needs to be improved. However, the nomogram for the prognosis 3 months after the operation has a very ideal prediction effect, which can well predict the poor prognosis 3 months after the operation. This is also the prognostic outcome that we are more concerned about.

## Figures and Tables

**Figure 1:** The cases selecting process.

**Figure 2:** The predictive nomogram and ROC curve and calibration curve of nomogram predicting the prognosis at 3 months after IVT. (a) Predictive nomogram of prognosis at 3 months after IVT; (b) the ROC curve of nomogram predicting the prognosis at 3 months after IVT in training cohort; (c) the ROC curve of nomogram predicting the prognosis at 3 months after IVT in verification cohort; (d) the calibration curve of nomogram predicting the prognosis at 3 months after IVT in training cohort; (e) the calibration curve of nomogram predicting the prognosis at 3 months after IVT in verification cohort. Note: In the calibration curve, the abscissa represents the predicted probability for the poor prognosis, and the ordinate represents the actual probability for the poor prognosis. “Apparent” indicates the predicted probability of the risk model for the whole queue; “Bias-corrected” indicates the predicted probability corrected by bias-corrected approach Bootstrapping; “Ideal” indicates the ideal predicted probability. The better the coincidence of the three indicators is, the better the prediction performance of the nomogram is.

**Figure 3:** The decision curve and clinical impact curve analysis of nomogram predicting the prognosis at 3 months after IVT. (a) The decision curve of nomogram predicting the prognosis at 3 months after IVT in training cohort; (b) the decision curve of nomogram predicting the prognosis at 3 months after IVT cohort; (c) the nomogram predicting the CICA of the prognosis at 3 months after IVT in training cohort; (d) the nomogram predicting the CICA of the prognosis at 3 months after IVT in verification cohort. Note: (1) In the decision curve, the abscissa represents the high-risk threshold probability to predict poor prognosis, and the ordinate represents net benefit. “Model” refers to the net benefit brought by intervention through predicting high-risk patients with poor prognosis under different threshold probabilities according to the risk model; “All” and “None” represent two extreme cases. “All” refers to the net benefit brought by intervention when all patients were at high risk with poor prognosis. “None” refers to no intervention when all patients were at low risk, and under this condition, the net benefit was 0. DCA was used to analyze and compare two extreme cases, the net benefit of the risk model and the corresponding threshold probability. (2) As to the CICA, we assumed that 1000 patients were applied to our model under simulated examination conditions. “Number high risk” represents the number of high-risk patients with poor prognosis predicted by the model at different threshold probabilities. “Number high-risk event” represents the actual number of high-risk patients with poor prognosis.

**Figure 4:** The predictive nomogram and ROC curve and calibration curve of nomogram predicting the early neurological recovery after IVT. (a) Predictive nomogram of early neurological recovery after IVT; (b) the ROC curve of the nomogram predicting the early neurological recovery after in training cohort; (c) the ROC curve of the nomogram predicting the early neurological recovery after in verification cohort; (d) the calibration curve of nomogram predicting the early neurological recovery after IVT in training cohort; (e) the calibration curve of nomogram predicting the early neurological recovery after IVT in verification cohort. Note: The calibration curve has been explained in Figure 2.

**Figure 5:** The decision curve and clinical impact curve analysis of nomogram predicting the early neurological recovery after IVT. (a) The decision curve of nomogram predicting the early neurological recovery after IVT in training cohort; (b) the decision curve of nomogram predicting the early neurological recovery after IVT in verification cohort; (c) the clinical impact curve of the nomogram predicting the early neurological recovery after IVT in training cohort; (d) the clinical impact curve of the nomogram predicting the early neurological recovery after IVT in verification cohort. Note: DCA and CICA have been explained in Figure 3.

**Table 1:** The prognosis of included cases.

Group	All (*N* = 849)	Training cohort (*N* = 594)	Verification cohort (*N* = 255)
Age	70.07 ± 12.54	70.12 ± 12.45	69.95 ± 12.77
Poor early neurological function recovery	452 (53.2%)	320 (53.9%)	132 (51.8%)
Poor prognosis at 3 months	294 (34.6%)	209 (35.2%)	85 (33.3%)

**Table 2:** The univariate analysis of prognosis of patients with ischemic stroke at 3 months after IVT.

No.	Factors	All (N = 594)	Group 1 (*N* = 209)	Group 0 (*N* = 385)	*t*/*z*/*χ*^2^	*P*
1	Gender (male)	337 (56.7%)	101 (48.3%)	236 (61.3%)	9.288	0.003
2	Ages (year)	70.12 ± 12.45	76.31 ± 11.06	66.76 ± 11.88	9.585	<0.001
3	BMI (kg/m^2^)	22.73 ± 3.52	21.96 ± 3.53	23.15 ± 3.44	-3.977	<0.001
4	BNIHSS (score)	5 (2.75, 12.00)	12 (7, 19)	3 (2, 7)	-12.688	<0.001
5	Smoking (yes)	173 (29.1%)	47 (22.5%)	126 (32.7%)	6.880	0.009
6	SecondThrombolysis (yes)	13 (2.2%)	5 (2.4%)	9 (2.1%)	0.630	0.820
7	Hypertension (yes)	409 (68.9%)	156 (74.6%)	253 (65.7%)	5.034	0.025
8	preAF (yes)	95 (16.0%)	55 (26.3%)	40 (10.4%)	25.574	<0.001
9	preIHD (yes)	36 (6.1%)	17 (8.1%)	19 (4.9%)	2.435	0.119
10	NewAF (yes)	28 (4.7%)	15 (7.2%)	13 (3.4%)	4.356	0.037
11	DM (yes)	89 (15.0%)	39 (18.7%)	50 (13.0%)	3.423	0.064
12	HL (yes)	18 (3.0%)	6 (2.9%)	12 (3.1%)	0.028	0.867
13	CHD (yes)	47 (7.9%)	20 (9.6%)	27 (7.0%)	1.215	0.270
14	CHF (yes)	17 (2.9%)	10 (4.8%)	7 (1.8%)	4.288	0.038
15	PreStrokeHistory (yes)	87 (14.6%)	42 (20.1%)	45 (11.7%)	7.659	0.006
16	CHDHistory (yes)	3 (0.5%)	1 (0.5%)	2 (0.5%)	0.005	0.946
17	HHcy (yes)	33 (5.6%)	14 (6.7%)	19 (4.9%)	0.803	0.370
18	Aspirin (yes)	77 (13.0%)	31 (14.8%)	46 (11.9%)	0.999	0.318
19	Clopidogrel (yes)	17 (2.9%)	10 (4.8%)	7 (1.8%)	4.288	0.038
20	Warfarin (yes)	8 (1.3%)	5 (2.4%)	3 (0.8%)	2.653	0.103
21	Atorvastatin (yes)	27 (4.5%)	9 (4.3%)	18 (4.7%)	0.043	0.837
22	Rosuvastatin (yes)	25 (4.2%)	14 (6.7%)	11 (2.9%)	4.958	0.026
23	PreSBP (mmHg)	154.81 ± 20.18	157.09 ± 19.58	153.57 ± 20.42	2.034	0.029
24	PreDBP (mmHg)	84.9 ± 12.72	84.14 ± 12.96	85.31 ± 12.59	-1.073	0.513
25	Hb (g/L)	139.41 ± 17.03	135.23 ± 18.96	141.68 ± 15.45	-4.214	<0.001
26	RBC (◊10^12^/L)	4.58 (4.26, 4.93)	4.46 (4.03, 4.84)	4.66 (4.35, 5.00)	-4.745	<0.001
27	WBC (◊10^9^/L)	7.65 ± 3.41	7.79 ± 2.99	7.57 ± 3.63	0.779	0.436
28	N (%)	63.01 ± 12.44	64.61 ± 13.2	62.14 ± 11.94	2.254	0.025
29	PLT (◊10^9^/L)	186.53 ± 58.31	181.31 ± 55.71	189.37 ± 59.55	-1.610	0.108
30	K+ (mmol/L)	3.76 ± 0.48	3.77 ± 0.5	3.75 ± 0.46	0.353	0.725
31	Na+ (mmol/L)	141.17 ± 4.3	141.11 ± 4.64	141.2 ± 4.11	-0.240	0.811
32	UN (mmol/L)	6.03 (4.90, 7.20)	6.30 (5.00, 7.70)	5.90 (4.90, 6.99)	-2.473	0.013
33	Cr (*μ*mol/L)	77.1 ± 26.35	79.64 ± 32.42	75.72 ± 22.3	1.556	0.121
34	PT (s)	11.43 ± 1.06	11.55 ± 1.17	11.37 ± 1.00	1.955	0.051
35	APTT (s)	30.22 ± 4.96	29.51 ± 4.92	30.61 ± 4.94	-2.609	0.009
36	INR	1 ± 0.09	1.01 ± 0.09	0.99 ± 0.09	2.498	0.013
37	Fg (g/L)	3.38 (2.69,4.03)	3.50 (2.77,4.22)	3.29 (2.65,3.88)	-2.754	0.006
38	Time (min)	154.7 ± 60.1	161.58 ± 61.75	150.97 ± 58.92	2.061	0.040
39	Drug (u-PA)	49 (8.2%)	25 (12.0%)	24 (6.2%)	5.872	0.015
40	24hNIHSS (score)	3 (1, 9)	11 (6, 22)	2 (1, 4)	15.251	<0.001

Note: Group 1 is poor neurological function recovery group, and group 0 is good neurological function recovery group.

**Table 3:** Logistic regression analysis on prognosis of patients with ischemic stroke at 3 months after IVT.

Factors	*B*	S.E.	Wald	*P*	OR	OR 95% CI	
						Low	Up
Ages (year)	0.048	0.011	18.792	0.001	1.050	1.027	1.073
DM (yes)	0.821	0.303	7.333	0.007	2.272	1.254	4.115
APTT (s)	-0.050	0.025	4.036	0.045	0.952	0.906	0.999
Drug (u-PA)	1.100	0.409	7.237	0.007	3.003	1.348	6.693
V24hNIHSS (score)	0.263	0.027	95.063	0.001	1.301	1.234	1.371
Constant	-5.603	1.113	25.328	0.001	0.004		

**Table 4:** Univariate analysis of early neurological recovery after IVT of patients with ischemic stroke.

No.	Factors	All (*N* = 594)	Group 1 (*N* = 320)	Group 0 (*N* = 274)	*t*/*z*/*χ*^2^	*P*
1	Gender (male)	337 (56.7%)	171 (53.4%)	166 (60.6%)	3.071	0.080
2	Ages (year)	70.12 ± 12.45	71.93 ± 12.35	68.01 ± 12.26	3.873	<0.001
3	BMI (kg/m^2^)	22.73 ± 3.52	22.38 ± 3.53	23.15 ± 3.46	-2.701	0.007
4	BNIHSS (score)	5 (2.75, 12.00)	6 (3, 13)	4 (2, 11)	-4.939	<0.001
5	Smoking (yes)	173 (29.1%)	94 (29.4%)	79 (28.8%)	0.021	0.885
6	SecondThrombolysis (yes)	13 (2.2%)	4 (1.3%)	9 (3.3%)	2.855	0.091
7	Hypertension (yes)	409 (68.9%)	232 (72.5%)	177 (64.6%)	4.297	0.038
8	preAF (yes)	95 (16.0%)	60 (18.8%)	35 (12.8%)	3.924	0.048
9	preIHD (yes)	36 (6.1%)	19 (5.9%)	17 (6.2%)	0.018	0.892
10	NewAF (yes)	28 (4.7%)	11 (3.4%)	17 (6.2%)	2.516	0.113
11	DM (yes)	89 (15.0%)	57 (17.8%)	32 (11.7%)	4.360	0.037
12	HL (yes)	18 (3.0%)	7 (2.2%)	11 (4.0%)	1.677	0.195
13	CHD (yes)	47 (7.9%)	28 (8.8%)	19 (6.9%)	0.668	0.414
14	CHF (yes)	17 (2.9%)	7 (2.2%)	10 (3.6%)	1.135	0.287
15	PreStrokeHistory (yes)	87 (14.6%)	50 (15.6%)	37 (13.5%)	0.531	0.466
16	CHDHistory (yes)	3 (0.5%)	1 (0.3%)	2 (0.7%)		0.598∗
17	HHcy (yes)	33 (5.6%)	21 (6.6%)	12 (4.4%)	1.341	0.247
18	Aspirin (yes)	77 (13.0%)	38 (11.9%)	39 (14.2%)	0.728	0.394
19	Clopidogrel (yes)	17 (2.9%)	11 (3.4%)	6 (2.2%)	0.827	0.363
20	Warfarin (yes)	8 (1.3%)	5 (1.6%)	3 (1.1%)		0.731∗
21	Atorvastatin (yes)	27 (4.5%)	18 (5.6%)	9 (3.3%)	1.863	0.172
22	Rosuvastatin (yes)	25 (4.2%)	12 (3.8%)	13 (4.7%)	0.362	0.547
23	PreSBP (mmHg)	154.81 ± 20.18	156.34 ± 19.16	153.02 ± 21.21	2.003	0.046
24	PreDBP (mmHg)	84.9 ± 12.72	84.91 ± 12.97	84.89 ± 12.44	0.015	0.988
25	Hb (g/L)	139.41 ± 17.03	138.51 ± 17.71	140.46 ± 16.17	-1.395	0.164
26	RBC (◊10^12^/L)	4.58 (4.26, 4.93)	4.54 (4.14, 4.89)	4.65 (4.35, 4.98)	-2.717	0.007
27	WBC (◊10^9^/L)	7.65 ± 3.41	7.86 ± 3.62	7.4 ± 3.14	1.629	0.104
28	N (%)	63.01 ± 12.44	64.16 ± 13.14	61.67 ± 11.45	2.462	0.014
29	PLT (◊10^9^/L)	186.53 ± 58.31	186.97 ± 59.26	186.02 ± 57.28	0.198	0.843
30	K+ (mmol/L)	3.76 ± 0.48	3.75 ± 0.48	3.76 ± 0.47	-0.339	0.735
31	Na+ (mmol/L)	141.17 ± 4.3	141 ± 4.15	141.36 ± 4.47	-0.999	0.318
32	UN (mmol/L)	6.03 (4.90, 7.20)	6.10 (4.93, 7.47)	6.00 (4.90, 7.00)	-0.924	0.355
33	Cr (*μ*mol/L)	77.1 ± 26.35	78.42 ± 30.5	75.56 ± 20.42	1.358	0.175
34	PT (s)	11.43 ± 1.06	11.4 ± 1	11.48 ± 1.14	-0.953	0.341
35	APTT (s)	30.22 ± 4.96	29.82 ± 4.95	30.7 ± 4.93	-2.157	0.031
36	INR	1 ± 0.09	0.99 ± 0.09	1 ± 0.09	-0.948	0.343
37	Fg (g/L)	3.38 (2.69, 4.03)	3.46 (2.73, 4.11)	3.30 (2.68, 3.91)	-1.681	0.093
38	Time (min)	154.7 ± 60.1	160.47 ± 60.24	147.96 ± 59.33	2.541	0.011
39	Drug (u-PA)	49 (8.2%)	36 (11.3%)	13 (4.7%)	8.254	0.004

Note: (1) Group 1 is the poor early neurological function recovery group; group 0 is the good early neurological function recovery group; (2) ^∗^*P* represents the *P* value calculated by Fisher's exact probability method.

**Table 5:** Multivariate logistic regression analysis of early neurological recovery after IVT in patients with ischemic stroke.

Factors	*B*	S.E.	Wald	*P*	OR	OR 95% CI	
						Low	Up
Ages (year)	0.022	0.007	8.654	0.003	1.022	1.007	1.037
BNIHSS (score)	0.029	0.011	6.492	0.011	1.030	1.007	1.053
DM (yes)	0.516	0.244	4.477	0.034	1.675	1.039	2.701
N (yes)	0.014	0.007	4.154	0.042	1.014	1.001	1.028
Drug (u-PA)	0.971	0.345	7.917	0.005	2.641	1.343	5.194
Constant	-3.535	0.762	21.524	0.001	0.029		

## Data Availability

The data that support the findings of this study are available from the corresponding author upon reasonable request.

## Supplementary Materials

Supplementary materials Table S1: comparison of the above-mentioned independent influencing factors in the two groups. Table S2: analysis of multiple factors affecting the prognosis of stroke patients after IVT.
